# Groundwater Quality: The Application of Artificial Intelligence

**DOI:** 10.1155/2022/8425798

**Published:** 2022-08-24

**Authors:** Mosleh Hmoud Al-Adhaileh, Theyazn H. H. Aldhyani, Fawaz Waselallah Alsaade, Mohammed Al-Yaari, Ali Khalaf Ahmed Albaggar

**Affiliations:** ^1^Al Bilad Bank Scholarly Chair for Food Security in Saudi Arabia, The Deanship of Scientific Research, The Vice Presidency for Graduate Studies and Scientific Research, King Faisal University, Al Ahsa 31982, Saudi Arabia; ^2^Deanship of E-learning and Distance Education King Faisal Unversity, P.O. Box 380, Al-Ahsa 31982, Saudi Arabia; ^3^Applied College in Abqaiq, King Faisal University, P.O. Box 400, Al-Ahsa 31982, Saudi Arabia; ^4^College of Computer Science and Information Technology, King Faisal University, P.O. Box 400, Al-Ahsa 31982, Saudi Arabia; ^5^Chemical Engineering Department, King Faisal University, P.O. Box 380, Al-Ahsa 31982, Saudi Arabia; ^6^Department of Biology, Faculty of Sciences and Arts in Baljurashi, Albaha University, PO. Box: 335, Zip Code: 22888, Al Bahah, Saudi Arabia

## Abstract

Humans and all other living things depend on having access to clean water, as it is an indispensable essential resource. Therefore, the development of a model that can predict water quality conditions in the future will have substantial societal and economic value. This can be accomplished by using a model that can predict future water quality circumstances. In this study, we employed a sophisticated artificial neural network (ANN) model. This study intends to develop a hybrid model of single exponential smoothing (SES) with bidirectional long short-term memory (BiLSTM) and an adaptive neurofuzzy inference system (ANFIS) to predict water quality (WQ) in different groundwater in the Al-Baha region of Saudi Arabia. Single exponential smoothing (SES) was employed as a preprocessing method to adjust the weight of the dataset, and the output from SES was processed using the BiLSTM and ANFIS models for predicting water quality. The data were randomly divided into two phases, training (70%) and testing (30%). Efficiency statistics were used to evaluate the SES-BiLSTM and SES-ANFIS models' prediction abilities. The results showed that while both the SES-BiLSTM and SES-ANFIS models performed well in predicting the water quality index (WQI), the SES-BiLSTM model performed best with accuracy (*R* = 99.95% and RMSE = 0.00910) at the testing phase, where the performance of the SES-ANFIS model was *R* = 99.95% and RMSE = 2.2941 × 100-07. The findings support the idea that the SES-BilSTM and SES-ANFIS models can be used to predict the WQI with high accuracy, which will help to enhance WQ. The results demonstrated that the SES-BiLSTM and SES-ANFIS models' forecasts are accurate and that both seasons' performances are consistent. Similar investigations of groundwater quality prediction for drinking purposes should benefit from the proposed SES-BiLSTM and SES-ANFIS models. Consequently, the results demonstrate that the proposed SES-BiLSTM and SES-ANFIS models are useful tools for predicting whether the groundwater in Al-Baha city is suitable for drinking and irrigation purposes.

## 1. Introduction

Water is the most crucial of all resources and is essential for the survival of all forms of life. Unfortunately, it is constantly threatened by pollution caused by the same things that support life. Water is one of the most communicative media available, and it has a long range. Correspondingly, rapid industrialization has resulted in an alarming decline in the quality of drinking water worldwide. The World Health Organization estimates that 3.57 million people each year lose their lives as a result of diseases that are associated with water [1]. It has been known for a very long time that one of the most significant factors contributing to the proliferation of terrible diseases is insufficient water quality. According to figures provided by the World Health Organization, water-related illnesses claim the lives of 3.57 million people every year [2]. For a long time, poor water quality has been identified as a major factor in the spread of deadly diseases. Schistosomiasis is an acute and chronic sickness caused by parasitic worms that can be transmitted through contact with contaminated water, according to the World Health Organization [2]. Diseases, including diarrhea, typhoid fever, gastroenteritis, cryptosporidium infections, and hepatitis, are the most common cause of these disorders. Typhoid bacteria are responsible for most of these illnesses. Fresh water is found in rivers and groundwater alike, and it accounts for only three percent of the entire water supply on the planet [3].

The Kingdom of Saudi Arabia (KSA) relies heavily on groundwater to meet its needs for drinking water and irrigation. Groundwater extraction in the KSA has expanded over the past three decades, reaching a total of 17 billion m^3^/year. Indeed, groundwater supplies 80% of the water requirements of the KSA [4]. Compared to the amount of water being drained each year, groundwater recharge is extremely low. The lowering of groundwater levels can also have a negative impact on the quality of the water [5]. The deep aquifers in the sedimentary strata that make up the Arabian shield have developed secondary porosities [6]. These porosities are located on top of the fractured Precambrian bedrock. There are also aquifers that are found, and while they are shallower than the valleys, they play a crucial role in the Arabian shields and coastal regions [7]. Agriculture was another industry that put a significant amount of weight on groundwater resources in the 1970s. Groundwater resources in an already water-stressed region have grown problematic in terms of both quantity and quality as a result of rapid urbanization, expanding industrial activity, and a growing population [8].

In addition, because of either anthropogenic or natural/geogenic causes, groundwater quality deteriorates [9]. Groundwater quality is a major concern in the study area due to local climatic and geological factors. The way in which water interacts with soils and sediments, the flow path, rock types, and common geochemical conditions such as dissolved oxygen, reduced oxygen, leaching, and ion exchange all have an effect on the quality of groundwater. These are just some of the many factors that influence groundwater quality [10]. Hence, water pollution is a serious problem in the KSA, harming the sustainability of water resources, which might create an insufficient water supply for all people, even when a great number of water resources are accessible [11].

Indeed, water is the most critical natural resource problem that humankind will have to handle in the 21st century. The combined consequences of human activity and climate change have resulted in considerable changes in runoff from numerous groundwater and growing water shortages. Water shortages not only present a danger to human life and social development but also have a considerable influence on the gross domestic product. To limit the effects of water pollution, the monitoring and evaluation of groundwater quality are vital [12].

The water quality index (WQI) provides decision makers with information that is crucial to their work. There is no common strategy for predicting and categorizing the WQI [13], though researchers have used the artificial intelligence (AI) method to address these difficulties [14]. AI-based modeling eliminates the need for subindex computations and delivers a WQI value in a short time. The AI technique, in addition, has the benefit of being less sensitive to missing values and being able to perform sophisticated mathematical calculations with a huge quantity of data and nonlinear structures. Many academics are paying close attention to the use of AI-based methodologies, such as machine learning, in their studies. A wide variety of works on machine learning models have been produced in the course of previous study. Some examples of these models include artificial neural networks, decision trees, *k*-nearest neighbors, Naive Bayes, and support vector machines. However, these typical machine learning approaches have several drawbacks, such as a high level of bias and overfitting [15]. Accordingly, machine learning algorithms that use ensemble approaches, such as bagging and boosting, to solve these challenges are being developed and improved [16]. Using ensemble models that combine the judgments of numerous base classifiers, more accurate predictions can be made. New machine learning techniques, such as gradient boosting [17] and the random forest approach [18–22], have been of great help in the prediction of water quality in recent years.

A number of research works have made use of ANN models in order to predict and anticipate the quality of the water. According to this body of research, ANNs are capable of reliably predicting the quality of drinking water. According to this work, the prediction and modeling of water quality are being improved by making use of a wide variety of cutting-edge technologies, such as fuzzy logic, stochastic, artificial neural networks (ANNs), and deep learning models [23, 24]. This is being done in order to better understand how water quality can be predicted and modeled.

An artificial neural network (ANN) model was developed by Palani et al. [25] for the purpose of forecasting DO, salinity, temperature, and chlorophyll-a concentrations in the coastal water of Singapore. The ANN model displayed an excellent correlation value of 0.8-0.9, as stated by Palani et al. ANFIS, the radial bias function, and multilayer sensory neural network models were utilized by Ahmed et al. [26] in order to estimate the ammoniacal nitrogen concentration of water samples. Wavelet data denoising was also utilized during this process. The authors discovered that removing noise from the data improved the performance of the prediction models. In order to estimate DO in sand media filters, Marti et al. [27] utilized ANN, GEP, and regression, which required a total of 769 data points derived from experimental results. The electrical conductivity, the pH, the amount of dissolved oxygen, and the head loss were the most useful parameters. Based on the findings, it was determined that the gene expression programming (GEP) model provided a more accurate estimation than the other approaches. The authors of this work estimated the total suspended solids (TSS), biochemical oxygen demand, chemical oxygen demand, and total dissolved solids (TDS) in a drainage basin by using a regression tree and support vector regression models. According to the authors, the support vector regression (SVR) fared better than the RT in terms of accurately predicting the desired output. Sarkar and Pandey [28] employed ANN to make predictions for DO. Accurate ANN results with a correlation coefficient close to 0.9 were reported by the authors. Support vector machine (SVM) and ANN methods were used by Haghiabi et al. [29] to predict various water quality indicators. Both ANN and SVM were shown to be effective in the prediction of water quality by the authors. To predict the capacity of a water treatment facility, Zhang et al. [30] employed a hybrid neural network model. The study's findings demonstrated that employing a larger dataset improved the model's performance. Shafi et al. [31] used support vector machines, neural networks (NN), and deep neural networks (DNN) for prediction of WQI. A total of 25 parameters were integrated as input parameters into single feedforward neural networks to identify water quality [32]. Dissolved oxygen (DO) was predicted using an ANN model developed by Rankovic et al. [33]. Gazzaz et al. [34] predicted the WQI using ANN models and Internet of Things (IoT) technologies. ANN and regression were utilized by Abyaneh [35] to predict the chemical oxygen requirements. Sakizadeh [36] estimated the water quality indicator using ANNs with Bayesian regularization (WQI). This sort of neural network (ANN) model, known as the radial basis function (RBF), has been used to predict and characterize water quality.

Moreover, deep learning has recently become more popular in water quality modeling. In a deep learning approach, neural network topologies typically include one input layer, many hidden layers, and a single output layer [37−39]. Liu et al. [40] used LSTM networks to develop a drinking water quality model for the Yangtze River basin. When they assessed the pH, DO, COD, and the content of ammonium nitrate (NH3-N), they found that the suggested LSTM network could be used to predict drinking water quality indicators. A hybrid convolutional neural network (CNN) LSTM model was proposed by Barzegar et al. [41] for the purpose of estimating the concentrations of DO and chlorophyll-a (Chl-a) in the Small Prespa Lake in Greece.

As a result, the purpose of this study is to develop an improved hybrid model by making use of models that incorporate single exponential smoothing with bidirectional long short-term memory (SES-BiLSTM) and single exponential smoothing adaptive neurofuzzy inference system (SES-ANFIS). This will allow the researchers to determine whether or not the groundwater in the Al-Baha region is suitable for drinking and irrigation. This study will be helpful in the identification, within a short amount of time, of the appropriateness of drinking water and irrigation water, particularly in arid and semidry regions. The major contribution to research that was made by this paper may be stated as follows.

The groundwater quality in the region of Al-Baha was evaluated using WQI values:

- An adaptive neurofuzzy inference system (SES-ANFIS) was developed, and a demonstration of the computing capability of single exponential smoothing (SES) with bidirectional long short-term memory (BiLSTM) was presented
- The suggested model's general framework was delineated for groundwater prediction
- The use of correlation coefficients was tested efficiently to find the best groundwater parameters
- An alternative technique, a neural network model, was developed to predict groundwater quality directly

## 2. Materials and Methods

### 2.1. The Study Area

In this work, water samples from 19 groundwater wells in the Al-Baha region of Saudi Arabia were collected. These wells have long served as the main source of drinking and irrigation water. The locations and altitudes of these wells are presented in Table 1. Subsequently, water samples were analyzed to obtain their physical, chemical, and bacterial properties (i.e., water quality data). These data include pH, total dissolved solids (TDS), turbidity, iron (Fe) concentration, manganese (Mn) concentration, sulfate (SO_4_^2−^) concentration, nitrate (NO_3_^−^) concentration, nitrite (NO_2_^−^) concentration, and the colony-forming unit (cfu) of coliform bacteria per 100 milliliters (ml). The details of the water sampling and analysis are reported elsewhere [42].

### 2.2. Water Quality Index and Classification

The water quality index (WQI) can be used to evaluate the water quality as per the measured values of some parameters affecting water quality. In this investigation, nine parameters, mentioned earlier, were measured and used for the WQI calculations as follows:

(1) $$\begin{array}{c} \text{WQI}=\frac{\sum_{i=1}^{N}q_{i}\times x_{i}}{\sum_{i=1}^{N}x_{i}}, \end{array}$$

where *N*, *q*_*i*_, and *x*_*i*_ are the number of parameters, the quality rating scale of each parameter, and the unit weight of each parameter, respectively. The following equations can be used to calculate *q*_*i*_ and *x*_*i*_:

(2) $$\begin{array}{c} q_{i}=100\times \left(\frac{P_{i}-P_{\text{Ideal}}}{S_{i}-P_{\text{Ideal}}}\right),\\ K=\frac{1}{\sum_{i=1}^{N}S_{i}},\\ x_{i}=\frac{K}{S_{i}}, \end{array}$$

where *P*_*i*_ and *P*_Ideal_ are the measured and ideal values of parameter *i*, respectively, and *S*_*i*_ is the KSA standard value of parameter *i*, as shown in Table 2.

The generic framework of the proposed system for prediction and classification of the water quality is presented in Figure 1.

### 2.3. Preprocessing Methods

#### 2.3.1. Min-Max Normalization

The Min-Max normalization was utilized in order to scale the input variables to a range that was comprised of zeros and ones. As part of the data preparation process for machine learning, data normalization is performed. Changing the values of input and output variables to a single scale is the purpose of normalization. For the normalization process, *x*_min_ and *x*_max_ are, respectively, the minimum and maximum values for the *i*^th^ attribute.

(3) $$\begin{array}{c} \overset{`}{x=\frac{x-x_{\min}}{x_{\max}-x_{\min}}}. \end{array}$$

For example, *x*_min_ is equal to the normalized value of the input variable *x*_*i*_ divided by the maximum input variable *x*_max_ and minimum variable *x*_min_.

#### 2.3.2. Single Exponential Smoothing (SES) Model

One of the statistical procedures that is used most frequently, known as the single exponential smoothing model, is used to anticipate data that does not have a trend and does not have seasonal variations. The model only uses the weighted observation data to obtain prediction data, and it only uses one significant parameter (alpha). The metrics of evaluation will guide the selection of appropriate values for these parameters:

(4) $$\begin{array}{c} \ell_{0}=\bar{X}=\frac{\sum_{t=1}^{n}Xy_{t}}{n},\\ P_{T+1}=\alpha y_{t}+\left(1-\alpha \right)P_{t}, \end{array}$$

*ℓ*_0_ is the level of trend, *X* is the level of trend, and *n* is the number of samples in the dataset. The output is *y*_*t*_. When smoothing out the training data, the alpha values are set to 0 on a scale of 10–1, 0 ≤ *α* ≤ 10 ≤ *α* ≤ 1.

### 2.4. Prediction Models

#### 2.4.1. Bidirectional Long Short-Term Memory (BiLSTM) Algorithm

Recurrent neural networks, often known as RNNs, are a special kind of neural network with the ability to acquire new knowledge over the course of time. RNNs can be broken down into several subtypes, one of which is called long short-term memory (LSTM) neural networks. These networks are able to acquire knowledge on long-term dependencies. Each and every RNN has the same core structure, which consists of repeating neural network modules that are coupled to one another [40, 42–44]. LSTM networks, which are used to store information and have this chained in a similar pattern, also use purpose-built memory cells to store the information; however, the repeating module in an LSTM has a distinct structure. As can be seen in Figure 2, an LSTM cell is composed of four distinct layers that are capable of interacting with one another.

There are two memory vectors (*h* and *C*) and cell activation matrices (*C*) in Figure 2, both of which have the same size as the hidden vector *h*. The logistic sigmoid function is *σ*. Tanh's function task is to keep the numbers in the range of −1 to 1. The RNN's internal structure, for example, a tanh layer, is based on a neuron. To protect and control the memory state, LSTM uses three switches: the input gate (*i*_*t*_), the output gate (*o*_*t*_), and the forgotten gate (*f*_*t*_), together with a memory cell as a gate. These switches have varying weights and will be weighted according to the input data. Afterward, each switch determines whether it is on or off.

To begin, you must decide which messages in memory cells, such as (5), should be eliminated. When the timing is *t*, the weight matrix is *W*, the output is *h*_*t*−1_, the input is *x*_*t*_ for time *t*, and the bias value is *b*_*f*_. The sigmoid layer converts these to values ranging from 0 to 1. For the final forgotten gate, *f*_*t*_ represents the output, while the value of 1 is reserved for exclusive use.

(5) $$\begin{array}{c} \text{Forget gate layer}:f_{t}=\sigma \left(W_{ef}X_{t}+W_{ef}h_{t-1}+W_{cf}C_{t-1}+b_{f}\right). \end{array}$$

The decision of which new messages to store in the memory unit and to split into two sections, adding temporary states and updating old states, needs to be made once more. The sigmoid layer determines which values require an update, and the tanh layer creates a vector that can be used to find new candidate values in (6) and (7). Weight matrix *W*_*i*_, *W*_*c*_ is updated in equation (6), which multiplies old state *C*_*t*−1_/*f*_*t*_ by new candidate value *i*_*t*_ (it will be in *C*_*t*_, *b*_*i*_, and *b*_*c*_) to determine whether to forget the message. The new candidate value *i*_*t*_ (it will be in the new state *C*_*t*_) is the bias value.

(6) $$\begin{array}{c} \text{Input gate layer}:i_{t}=\sigma \left(W_{xi}X_{t}+W_{hi}h_{t-1}+W_{ci}C_{t-1}+b_{i}\right), \end{array}$$

(7) $$\begin{array}{c} \text{New memory cell}:C_{t}=\sigma \left(f_{t}c_{t-1}+i_{t}\tanh\left(W_{xc}X_{t}+\;W_{hc\;}h_{t-1}+b_{c}\right)\right). \end{array}$$

Equations (6) and (7) use a sigmoid layer to determine which sections of the memory unit need to be outputted, and the state of memory unit is passed on in the final decision of the output message. To get the output, multiply *o*_*t*_ by tanh (*C*_*t*_) and then by *h*_*t*_ after the tanh layer is applied. This value lies between -1 and 1, depending on the temperature. The bias value is *b*_0_.

(8) $$\begin{array}{c} \text{Output gate layer}:o_{t}=\sigma \left(W_{xo}X_{t}+W_{ho}h_{t-1}+W_{co}C_{t-1}+b_{o}\right),\\ h_{t}=O_{t}\times \;\tanh\left(C_{t}\right). \end{array}$$

The BiLSTM network is shown schematically in Figure 3. Each training sequence in the BiLSTM model contains two circulating neural networks, one backward and one forward, each connected to a single output layer. The model receives and exports training materials in both ways. Two RNNs are used to determine the final output based on the status of both RNNs' hidden layers, which are connected to each other via an output layer.

ANFIS is a well-known hybrid AI model that combines artificial neural networks and fuzzy logic (FL). It was first proposed by Jang in the 1990s. Fuzzification, rule, normalization, defuzzification, and aggregation are the five main layers of the ANFIS architecture. It has been demonstrated that neural networks are capable, when given such a framework, of deducing the parameters of the FL algorithm [43]. The ANFIS fuzzy inference system makes use of Takagi-Sugeno if-then rules, together with an appropriate membership function. As with ANN, hybrid ANFIS may also detect nonlinear relationships between inputs and outputs. Several studies, such as those in [45–49], have shown that ANFIS has a higher prediction efficiency than individual ANNs or FL. As a sort of artificial neural network, the ANFIS system relies on the Takagi-Sugeno fuzzy inference system, which combines the advantages of ANN and fuzzy logic in one framework.

(9) $$\begin{array}{c} \text{Rule}1:\text{if }x\text{ is }A_{1}\text{ and }y\text{ is }B_{1},\text{then }f_{1}=p_{1}x+q_{1}y+r_{1},\\ \text{Rule}1:\text{if }x\text{ is }A_{2}\text{ and }y\text{ is }B_{2},\text{then }f_{1}=p_{2}x+q_{2}y+r_{2}, \end{array}$$

where *A*_1_ and *B*_1_ represent the fuzzy sets and *p*_1_, *p*_2_, *q*_1_, *q*_2_, and *r*_1_ represent the subsequent parameters that are used to determine their values during the training stage. The five layers are fuzzification, inference, normalization, outcome, and output. There are five layers in ANFIS's architecture: inference, normalization, outcome, and output.  Figure 4 depicts these layers:

*Layer 1.* Each node in the “premise parameters” layer generates a “fuzzy membership degree” as a result of the parameters in this layer. In the first-level iteration, assume that *O*_1,*i*_ is its *i*^th^ level and *j*^th^ node.
  (10) $$\begin{array}{c} O_{1,i}=\mu A_{i}\left(x\right),\;\text{for }i=1,2, \end{array}$$
  (11) $$\begin{array}{c} O_{1,i}=\mu B_{i}\left(y\right),\;\text{for }i=1,2, \end{array}$$
  (12) $$\begin{array}{c} \mu \;A_{i}\left(x_{1}\right)=\frac{1}{1+{\left({\left(x-c\right)}_{i}/\sigma_{i}\right)}^{2b_{i}}}. \end{array}$$
In equations (10) and (11), the fuzzy membership functions *μ* *A*_*i*_(*x*) and *μ* *B*_*i*_(*y*) are used (MF). The fuzzy sets are represented by *A*_*i*_ and  *B*_*i*_. The formula for the Gaussian MF (GMF) is based on a Sugeno-type fuzzy inference system, where *x* and *σ*_*i*_ refer to the average and variance of the GMF, respectively.
*Layer 2.* The firing strength of each rule is calculated by multiplying the values of the nodes in the second layer:
  (13) $$\begin{array}{c} O_{2,i}=w_{i}=\mu A_{i}\left(x\right)*\mu B_{i}\left(y\right),\;\;i=1,2. \end{array}$$
*Layer 3.* As stated above, the primary goal of this layer is to compute *O*_3,*i*_ normalization:
  (14) $$\begin{array}{c} O_{3,i}=\bar{w_{i}}=\frac{w_{i}}{w_{1+w_{2}}}\;i=1,2. \end{array}$$
In this case, *O*_3*,i*_ is the output of layer 3, and, $\bar{w}$ is the inference system rules' normalized firing strength.
*Layer 4*. This layer has nodes that may adapt. It allows the adaptive nodes to be customized through the use of three parameters.
  (15) $$\begin{array}{c} O_{4,i}=\bar{w_{i}}.f_{i}=\bar{w_{i}}.\left(p_{i}x+q_{i}y+r_{i}\right), \end{array}$$
where *p*_*i*_,  *q*_*i*_, and *r*_*i*_ are the parameters of the inference system in the form of *O*_4,*i*_ of layer 4.
*Layer 5.* This is the inference layer, and its purpose is to produce the overall output by using the information from the layers that came before it.
  (16) $$\begin{array}{c} O_{5,i}\text{overall output}=\sum \bar{w_{i}}f_{i}=\frac{{\sum_{i}\bar{w_{i}}f}_{i}}{\sum_{i}w_{i}}. \end{array}$$

The topology of ANFIS model is presented in Figure 5.

For the purpose of predicting water quality, we have developed a prediction system that combines the single exponential smoothing (SES) algorithm with the bidirectional long short-term memory (SES-BiLSTM) algorithm and an adaptive neurofuzzy inference system (SES-ANFIS). The output from the single exponential smoothing (SES) algorithm was then processed by the LSTM and ANFIS models. This was the first step in the procedure. The development process is depicted in the flowchart shown in Figure 6.

### 2.5. Performance Measurement

The mean square error (MSE), root-mean square error (RMSE), mean absolute error, and coefficient of correlation are the metrics that are utilized in the analysis of artificial intelligence models for the forecasting of WQ (CC). The definitions of the metrics are as follows.

#### 2.5.1. Mean Square Error (MSE)

The estimator mean square error (MSE) quantifies the average square of the errors, that is, the average square of the difference between the observation's values *y*_*i*,observ_ and estimated values *y*_*i*, estim_.

(17) $$\begin{array}{c} \text{MSE}=\frac{1}{n}\sum_{i=1}^{n}{\left(y_{i,\text{observ}}-y_{i,\text{estim}}\right)}^{2}. \end{array}$$

#### 2.5.2. Root-Mean Square Error (RMSE)

The RMSE value indicates a better fit between observations *y*_*i*,observ_ and estimated values *y*_*i*, estim_, divided by number of observations (*n*).

(18) $$\begin{array}{c} \text{RMSE}=\sqrt{\sum_{i=1}^{n}\frac{{\left(y_{i,\text{observ}}-y_{i,\text{estim}}\right)}^{2}}{n}}. \end{array}$$

#### 2.5.3. Coefficient of Correlation (CC)

Coefficient (*r*) goes from -1 to 1 and reflects the weight of the correlation between observations and prediction. The closer you get to zero, the less linear the relationship between observations and predictions becomes. The strong negative linear relationship between -1 and 1, for example, is represented by the number zero, while the strong positive linear relationship between the number 1 and the number 0 is represented by the number one.

(19) $$\begin{array}{c} R\%=\frac{n\left(\sum_{i=1}^{n}y_{i,\text{observ}}\;\times y_{i,\text{estim}}\right)-\left(\sum_{i=1}^{n}y_{i,\text{observ}}\right)\left(\sum_{i=1}^{n}y_{i,\text{estim}}\right)}{\sqrt{\left[n{\left(\sum_{i=1}^{n}y_{i,\text{observ}}\right)}^{2}-{\left(\sum_{i=1}^{n}y_{i,\text{observ}}\right)}^{2}\right]\left[n{\left(\sum_{i=1}^{n}y_{i,\text{estim}}\right)}^{2}-{\left(\sum_{i=1}^{n}y_{i,\text{estim}}\right)}^{2}\right]}}\times 100. \end{array}$$

## 3. Experiment

Improvements to the LSTM and ANFIS models, the SES preprocessing method, were applied in this study for predicting water quality. The LSTM and ANFIS models were used to forecast water quality characteristics in groundwater in Al-Baha region. When developing the model, the training phase utilized seventy percent of the data, while the testing phase made use of thirty percent of the data. MATLAB 2020 was used to perform the analysis on the data. In order to carry out the simulation, we made use of a computer that had an Intel i7 processor and 8 gigabytes of random access memory.

### 3.1. Training Process

It is a collection of data samples that are utilized in the process of fitting the parameters of a prediction model to the training of observational data regarding the water quality. It is a necessary part of all ANNs models, and its inclusion enables these models to produce accurate forecasts or do the functions that are required of them. In this investigation, a training process consisting of seventy percent of the dataset has been used in order to validate the effectiveness of the LSTM and ANFIS models. This study made use of three distinct model efficiency statistics. These statistics were the mean square error (MSE), the root-mean square error (RMSE), and the standard deviation of the mean square error (SDME). These statistics were used to measure how far the actual values deviated from the expected values.  Table 3 shows the results of the proposed models at training phase for predicting water quality. In addition, the SES-ANFIS model has achieved very low values of MSE = 2.2941 × 100^−07^ and RMSE = 0.000478.

Figure 7 demonstrates that there is a perfect match between the observed values and the prediction values of water quality. This was accomplished by plotting the developing system along the *y*-axis and the experimental values along the *x*-axis. The SES-ANFIS model has achieved *R* value of 100%, while the SES-BiLSTM model has achieved *R* value of 99.82%.

In the training stage, the predicted values' histogram error is shown in Figure 8. Metrics such as the error histogram may be used to identify discrepancies between the expected and observation values. These error numbers might be negative, since they indicate how the prediction values differ from the training target values. An error of SES-ANFIS model is 0.00069, where error histogram of SES-BiLSTM is 0.001691.

### 3.2. Testing Process

Testing phase is utilized in the process of selecting the model's parameters, whereas test set is utilized in the process of evaluating the effectiveness of the model on an unexplored (real world) dataset. 30% of the dataset was considered as testing for validating the SES-BiLSTM and SES-ANFIS models for predicting water quality.  Table 4 shows the results of SES-BiLSTM and SES-ANFIS models for predicting WQ. The results have revealed that the developing system SES-BiLSTM and SEE-ANFIS models were successfully predicting. It is observed that the two models were found to be capable of predicting the groundwater with great accuracy. According to the MSE metric, the SES-ANFIS model has achieved much less prediction (MSE = 2.2941 × 100^−07^).

The WQ values that were predicted are depicted as a regression plot in Figure 9, which is used throughout the testing phases. In order to determine the degree of correlation that exists between the projected values and the actual values, Pearson's correlation is used in this graphic. The numbers along the *x*-axis represent the experimental data, while the values along the *y*-axis represent the prediction values generated by the SES-BiLSTM and SES-ANFIS models. Both models have been proved to have earned the same score, which is 99.95%.

The error histogram of the proposed system's SES-BiLSTM and SES-ANFIS models at testing phase is presented in Figure 10. The error histogram metrics are used to compute the error between the testing observation values and testing target values at 30 bins. It is observed that the error histogram of SES-ANFIS is 5.44 × 10^−06^ and the error histogram of SES-BiLSTM is 2 × 10^−05^.

Therefore, there is a good correlation between the predictions generated by the model and the actual data, which implies that SES-ANFIS and SES-BiLSTM models may be made with confidence, and this information can be utilized to develop laws and procedures to safeguard water sources.

### 3.3. Selective Analysis for Finding Significant Parameters

Many engineering and scientific sectors are adopting sensitivity analysis, which encompasses nearly all data processing and computational modeling and process simulation operations. A good indicator for the quantitative and qualitative management of surface water resources in arid and semiarid environments can be found in the upstream discharge planning of regulated groundwater and the relationship between water quality measures. The correlation coefficient method was applied to examine the effectiveness of inputs parameters, namely, pH, TDS (mg/l), turbidity (NTU), Fe (mg/l), Mn (mg/l), SO_4_^2−^ (mg/l), NO_3_^−^ (mg/l), and NO_2_^−^ (mg/l) with WQ parameter for predicting water quality. For each of these eight water quality factors, the input parameter's percentage effect may be shown in Figure 11. As an example, PH, NO_2_^−^ (mg/l), NO_3_^−^ (mg/l), TDS (mg/l), and SO_4_^2−^ (mg/l) were the most important input characteristics for predicting groundwater in Al-Baha region. NO_2_− (mg/l) and pH have scored the highest percentages of *R*: 100% and 95.59%, respectively.

## 4. Results and Discussion

The modeling and prediction of water quality have played a vital and substantial role in the reduction of the amount of time as well as the number of resources that are necessary for laboratory analysis. The use of artificial intelligence algorithms as a potential replacement for more traditional approaches to estimating and forecasting water quality was investigated. The case study was conducted in Al-Baha region, Saud Arabia, including groundwater.

Using our technology, we are certain that we can keep a close eye on both the water supply and the wastewater stream. It is our goal to create a real-time system and test an alternate way utilizing a sophisticated artificial intelligence model for accurately predicting and classifying water quality. To correctly replicate water levels and quality, this study recommends using a combination of the artificial intelligence techniques presented in this study. In this way, a more sustainable and effective approach to water management and sustainability can be developed. Our model has performed well when it comes to analyzing contaminants with the bare minimum of parameters. There was a total of eight parameters included in the dataset. In addition, we have determined that the four following factors are extremely important: PH, NO_2_− (mg/l), NO_3_^−^, and SO_4_^2−^.  Table 5 provides a summary of the findings of the existing models in comparison to our suggested system. Several of the research works that have been conducted have utilized machine learning models for the purposes of modeling and predicting.

According to the article, the SES-BiLSTM and SES-ANFIS models may be used to predict water quality and can be used in the development and implementation of integrated water protection systems, as well as in the implementation of sound environmental management practices. The SES-BiLSTM and SES-ANFIS techniques have various advantages over the computational approach in forecasting WQI.

This study attempted to prove that the SES-BiLSTM and SES-ANFIS models are effective tools for forecasting water quality and may be used to construct integrated water protection systems while applying appropriate environmental management practices. The proposed models have several advantages over the computational approach when it comes to forecasting WQI. A minimum of four different water quality measures must be calculated and then transformed into partial indications to use the second technique. The WQI is calculated using a formula that relies heavily on subindices. As a result, implementing an existing ANN model based on raw data is substantially simpler because no new calculations are required. To develop the model, certain water quality characteristics are needed, minimizing the cost of water quality monitoring, among other things.

## 5. Conclusion

In groundwater studies, one of the most difficult problems to solve is the prediction of groundwater level (GWL) using geoelectric characteristics. This is due in part to the fact that an empirical relationship between the level of groundwater and the geoelectric parameters has not been established yet. In this study, an effort was made to circumvent these obstacles by investigating the capacity of advance artificial neural networks (ANNs) to simulate nonlinear systems:

- The artificial intelligence models were designed to forecast and categorize the quality of drinking water by utilizing data from groundwater gathered in a variety of places in Al-Baha region. The goal of the models was to improve water quality for human use. WQI was used to determine the values of eight significant parameters: pH, TDS (mg/l), turbidity (NTU), Fe (mg/l), Mn (mg/l), SO_4_^2−^ (mg/l), NO_3_^−^ (mg/l), and NO_2_^−^ (mg/l). These were regarded as important factors for determining the quality of the water. Developing new methods that make use of more advanced SES-BiLSTM and SES-ANFIS algorithms is one way to contribute to the preservation of a secure environment.
- In the SES-ANFIS and SES-BiLSTM models, the correlation coefficient was found to be 99.95%, and the MSE was found to be equivalent to 2.2941 × 100^−07^ for testing. The suggested model was used to generate these findings, and the set was divided as follows: 70% was used for training, and 30% was used for testing. The SES-ANFIS and SES-BiLSTM models that were proposed in this paper have several benefits, one of which is the ease with which groundwater pollution levels can be evaluated. In addition, making use of these models makes it possible to skip the time-consuming calculations that are a part of the conventional WQI that is most commonly used.
- In further research, the authors want to try to accurately anticipate the quality of the water by making use of indications that are dependent on the location of the various pollution sources.
- The authors plan to discuss evaluating the quality of groundwater in further articles; in doing so, they hope to make use of more machine learning strategies. The findings that were achieved via the use of various approaches will be compared, and the influence that these methods have on the quality of the prediction will be studied. The limitation of this proposed work is using small datasets; therefore, we did not apply classification algorithms for categorizing the types of water.

## Figures and Tables

**Figure 1:** A generic framework.

**Figure 2:** LSTM model.

**Figure 3:** BiLSTM structure algorithm.

**Figure 4:** Structure of ANFIS model for predicting WQ.

**Figure 5:** Topology of ANFIS system for predicting WQ.

**Figure 6:** Flowchart of developing system. (a) SES-ANFIS; (b) SES-BiLSTM model.

**Figure 7:** Regression plot of the proposed system: (a) SES-ANFIS model and (b) SES-BiLSTM model at training process.

**Figure 8:** Histogram plot of the proposed system: (a) SES-ANFIS model and (b) SES-BiLSTM model at training process.

**Figure 9:** Regression plot of the proposed system: (a) SES-ANFIS model and (b) SES-BiLSTM model at testing process.

**Figure 10:** Histogram plot of the proposed system: (a) SES-ANFIS model and (b) SES-BiLSTM model at testing process.

**Figure 11:** Important parameters.

**Table 1:** Details of the targeted wells.

Location	No. of wells	Altitude (m)	Latitude	Longitude
Mudailif	1	47	19.534829	41.050467
Bani Dabian	6	2.410	19.963037	41.503160
		2.393	19.965565	41.514047
		2.313	19.966935	41.490027
		2.304	19.970397	41.499260
		2.275	19.971517	41.495268
		2.133	19.995739	41.535219
Southeast of Al-Baha	3	612	19.702417	41.700848
		1.785	19.739621	41.926028
		1.624	19.865282	41.927247
East of Al-Baha	3	1.906	19.994561	41.660098
		1.866	20.097328	41.585645
		1.857	20.101866	41.580797
Baljurashi	3	2.026	19.851837	41.604840
		2.027	19.854214	41.564965
		2.037	19.859957	41.549216
Al-Mandag	2	2.224	20.107243	41.426129
		2.189	20.108782	41.288857
		2.151	20.123787	41.288205

**Table 2:** Parameters' standard values according to the Saudi standards [42].

Parameters	*S *_*i*_
pH	7.5
TDS, mg/l	500
Turbidity, NTU	1
Fe concentration, mg/l	0.3
Mn concentration, mg/l	0.4
SO_4_^2−^ concentration, mg/l	250
NO_3_^−^ concentration, mg/l	50
NO_2_^−^ concentration, mg/l	0.2
Coliform bacteria, cfu/100 ml	100

^*∗*^Values of the Saudi standards are less than or equal to the WHO standards.

**Table 3:** Results of the proposed model at training process.

Models	MSE	RMSE	*R* (%)
SES-BiLSTM	0.00707	0.0841	99.82
SES-ANFIS	7.8088 × 10^−08^	0.000279	100

**Table 4:** Results of the proposed model at testing process.

Models	MSE	RMSE	*R* (%)
SES-BiLSTM	0.00910	0.0954	99.95
SES-ANFIS	2.2941 × 100^−07^	0.000478	99.95

**Table 5:** Comparison results between the proposed system and existing systems.

Reference	Years	Input parameters	Results	Models	Types of water
Ref. [50]	2021	pH, T-Alk, T-hard, DO, TS, MPN	*R* = 0.999 MRE = 0.775	Feedforward back-propagation	Drinking water
Ref. [44]	2021	DO, pH, EC, BOD, N-NO_3_, fecal coliform, total coliform	*R* = 96.1% RMSE = 0.0029	ANFIS	Drinking water India
Ref. [51]	2021	TDS, N-NO^2+^, N-NO_3_^−^, Ca, Mg, Na, K, Cl^−^, SO_4_^2−^, CO_3_^2−^, HCO_3_^−^, F^−^, pH, TH, SAR, RSC	RMSE = 0.057 testing RMSE = 0.066 training	ANN	Drinking water India
Ref. [52]	2021	pH, DO, BOD, turbidity, TS	MSE = 2.08 *R* = 99.07% testing	ANN	River India
Ref. [53]	2020	pH, WT, OS, TDS, NTU, N-NO_3_, P-PO_4_, BOD5, COD, Cl−	RMSE = 0.007 *R*^2^ = 81.01% testing RMSE = 0.009 *R*^2^ = 92.09 training	Multilayer perceptron neural networks	River (Algeria)
Ref. [54]	2016	DO, BOD, COD, pH, SS, N-NH3	*R * ^2^ = 98.01 RMSE = 1.598	ANN	Water river (Malaysia)
Ref. [34]	2012	pH, EC, TDS, NTU, WT, BOD, DO, N-NH3, Mg, Cl, F, TH, Fe, Zn, As, total coliform bacteria, *E. coli* bacteria, SS, N-NO_3_,	RMSE = 1.633 *R* = 0.977	Artificial neural network	River (Malaysia)
Proposed system SES-ANFIS	2022	PH, TDS (mg/l), turbidity (NTU), Fe (mg *i*-1), Mn (mg *i*-1), So_4_ (mg *i*-1), No_3_ (mg *i*-1), and NO_2_ (mg *i*-1)	MSE = 7.8088 × 10^−08^ RMSE = 0.000279 *R* = 100% at training MSE = 2.2941 × 100^−07^ RMSE = 0.000478 *R* = 99.95%	SES-ANFIS	Groundwater Saud Arabia

## Data Availability

The dataset is collected from https://bbrc.in/assessment-of-water-quality-in-some-wells-in-albaha-region-and-its-surrounding-area-saudi-arabia/.
